The article "Impact of Activation, Optimization, and Regularization Methods on the Facial Expression Model Using CNN" was retracted in 2023. Reasons: signs of a paper mill; compromised peer review; unreliable results or conclusions.

# Impact of Activation, Optimization, and Regularization Methods on the Facial Expression Model Using CNN

**DOI:** 10.1155/2022/3098604

**Published:** 2022-06-16

**Authors:** Irfan Ali Kandhro, Mueen Uddin, Saddam Hussain, Touseef Javed Chaudhery, Mohammad Shorfuzzaman, Hossam Meshref, Maha Albalhaq, Raed Alsaqour, Osamah Ibrahim Khalaf

**Affiliations:** ^1^Department of Computer Science, Sindh Madressatul Islam University, Karachi, Pakistan; ^2^College of Computing and IT, University of Doha for Science and Technology, Doha, Qatar; ^3^Department of Information Technology, Hazara University, Mansehra 21120, KP, Pakistan; ^4^National University of Modern Languages, Islamabad, Pakistan; ^5^Department of Computer Science, College of Computers and Information Technology, Taif University, Taif 21944, Saudi Arabia; ^6^Department of Information Technology, College of Computer and Information Sciences, Princess Nourah Bint Abdulrahman University, P.O. Box 84428, Riyadh 11671, Saudi Arabia; ^7^Department of Information Technology, College of Computing and Informatics, Saudi Electronic University, 93499, Riyadh, Saudi Arabia; ^8^Al-Nahrain University, Al-Nahrain Nanorenewable Energy Research Center Baghdad, Baghdad, Iraq

## Abstract

When it comes to conveying sentiments and thoughts, facial expressions are quite effective. For human-computer collaboration, data-driven animation, and communication between humans and robots to be successful, the capacity to recognize emotional states in facial expressions must be developed and implemented. Recently published studies have found that deep learning is becoming increasingly popular in the field of image categorization. As a result, to resolve the problem of facial expression recognition (FER) using convolutional neural networks (CNN), increasingly substantial efforts have been made in recent years. Facial expressions may be acquired from databases like CK+ and JAFFE using this novel FER technique based on activations, optimizations, and regularization parameters. The model recognized emotions such as happiness, sadness, surprise, fear, anger, disgust, and neutrality. The performance of the model was evaluated using a variety of methodologies, including activation, optimization, and regularization, as well as other hyperparameters, as detailed in this study. In experiments, the FER technique may be used to recognize emotions with an Adam, Softmax, and Dropout Ratio of 0.1 to 0.2 when combined with other techniques. It also outperforms current FER techniques that rely on handcrafted features and only one channel, as well as has superior network performance compared to the present state-of-the-art techniques.

## 1. Introduction

According to everyone's common knowledge, the advancement of computer technology has greatly facilitated the advancement of various sectors, including artificial intelligence and pattern classification [1]. In order to achieve a natural connection, there must be an amicable relationship between the human and the machine. Mehrabian [2] found that facial emotions carry 55% of the useful information incommunication, whereas sound and language convey just 38% and 7%, respectively, of this information. As a result, facial expressions convey a great deal of emotional information. Facial emotion recognition has been investigated extensively in the past few decades, and it has gained more and more scholars' attention in the process [3–6].

When it comes to nonverbal communication, facial expression recognition is a powerful tool for conveying emotions, states, and intentions. Numerous studies have been undertaken on autonomous facial expression in sociable robotics, data analytics, human-computer vision, medical therapy, and driver fatigue surveillance because of its significance. Automated FER has since been extensively examined and used to encode facial expression characteristics [7–9]. Indeed, it is possible to tackle the challenge by identifying basic expressions under regulated conditions, such as fontal faces and side pose emotions. There were six basic emotions described in the twentieth century by Ekman and Friesen based on cross-cultural research [10]. In psychology, the term “basic expression” refers to a set of facial expressions that can be used to indicate a wide range of human emotions. Advances in neuroscience and psychology have shown that these six emotions are culturally specific rather than universally applicable [11].

There are still problems with the action coding system and continuous approach when it comes to describing emotions in real-world situations [12–15]. The effect model, on the other hand, does not show how complex or sensitive our effective displays are. Complexity and changes in head pose, lighting, and occlusion are to bear responsibility. People have different ways of expressing themselves, and the background brightness and background color, the position of the image, and many other factors can all change the way an image is analyzed. The fact that unposed expressions are often subtle also affects how the image is analyzed. So, the reliable automated FER system is very important in the applications [16, 17].

The performance, speed, and intelligence requirements of traditional machine learning algorithms can no longer be met in the age of big data. This is especially true in the domains of identification, classification, and target detection, where deep learning has showed exceptional information processing abilities to get better at classification and prediction in the long term, deep learning can develop more abstract high-level features and attribute information [18]. Image features can be consistently extracted using the convolutional neural network (CNN) [19], which is a deep learning architecture. It has been widely used both in academic circles and in actual business applications, especially in the field of computer vision [20–27].

Comprehensive surveys on automatic expression analysis have been published in recent days. These surveys have focused on and established a set of standard algorithms for automated facial expression [28]. The convolutional neural network (CNN) has enabled significant performance in related tasks [29–32]. Current studies extensively use CNN methods to analyze various features and extract essential details from facial expressions while evaluating different datasets [31, 33]. These works differ considerably in terms of the CNN structure, preprocessing, training, testing, and validating protocols. Furthermore, it is not plausible to compare the model's performance in a single experiment based on the reported results found on existing issues and bottlenecks in existing CNN architectures, consequently increasing the FER model's performance.

The followings are some of our significant contributions:

- We focused on the performance of the facial expression recognition model on optimization, regularization, and activation parameters by reviewing the existing convolutional neural network-based methods.
- We compare convolutional neural network methods by highlighting the differences empirically under consistent settings.
- Moreover, based on this, we identified the dodgeand directions for improving the model's performance.
- Eventually, we confirm rationally that overcoming issues such as bottlenecks enhances the performance significantly.
- The proposed convolutional neural network architecture model achieves state-of-the-art facial expression recognition as shown in experiments performed on various datasets.

This paper is divided into the following section. Section 1 describes an introduction about the research being done. Section 2 discusses the related work where past and present FER techniques have been discussed. Section 3 describes the proposed FER model with a detailed description of various components. The experimental results are discussed in Section 4, and Section 5 concludes the paper.

## 2. Related Work

For its superior performance in image processing, computer vision, and image classification, the CNN approach has been widely adopted in deep learning for these applications. A halftone image classification and image processing system, developed by Zhang et al. [34], was built to assess significant aspects of videos/images, and it performed exceptionally well. Unsupervised learning was used to extract features from halftone images, and he proposed using stacked sparse autoencoders (SAE). According to Khorrami et al. [35], it is possible to get good results from CNN if they are taught to look at a face and determine which elements influence CNN's predictions. An initial step is to train a zero-biased CNN using facial expression data, which the authors use the expanded Cohn-Kanade (CK+) dataset and the Toronto Face Dataset as benchmarks. They next perform a qualitative examination of the network, observing the spatial patterns that most intensely stimulate the different types of neurons in the convolutional layers and show how they mimic facial action units (FAUs). A final step in this process is to verify that all FAUs visible in filter visualization correlate with facing movements in the CK + dataset. A flexible hypothesis pooling approach for image multiclassification was developed by Wei et al. [36]. The model accepts any number of object segment assumptions made about the object as the input. Each hypothesis was linked to a shared CNN in a step-by-step fashion. Finally, the model varied hypothesis outcomes are averaged with max pooling, resulting in classic predictors for multilabel predictions that are based on classic predictors. Face alignment, face detection, and face recognition are only a few of the issues in FER-related applications, among others. Characters can now express themselves in human expressions, thanks to a new method developed by Aneja et al. [37]. It begins with a training phase in which two CNNs are trained to recognize human and stylized character expressions. After that, they develop a shared embedding feature space by employing a technique called transfer learning. This involves learning the mapping between characters and persons. This embedding additionally enables the retrieval of pictures based on human expressions as well as pictures based on character expressions. To obtain human-like character expressions, the authors used a perceptual model. Finally, the authors use the newly acquired stylized character expression dataset to evaluate their method on various retrieval tasks. The authors also give evidence that the ranking order of the proposed attributes has a strong correlation with the ranking order that was provided by an expert on facial expressions and mechanical Experiments.

Li et al. [38] developed a CNN-based cascade model with a robust discriminative capability to maintain high performance while dealing with the problem of changes in visual properties due to changes in expressions, pose, and lighting in original face recognition. A deep learning model for face adjustment and alignment with landmark characteristics and recurrent recognition has been proposed by Parka et al. [39]. Chen et al. [40] use deep learning to demonstrate an effective method for recognizing smiles in the wild. Unlike previous works that collected handcrafted features from face pictures and trained a classifier to undertake smile detection in a two-step process, deep learning may be able to merge feature learning and classification into a single model rapidly. The authors use the deep convolutional network to overcome this popular deep learning model. Smile CNN is a deep convolutional network created by the authors to feature learning and smile detection simultaneously. Although a deep learning model is typically designed to handle “big data,” experimental results show that the model can also effectively manage “small data.” They are now looking at the discriminative power of the learned features, which are derived from the cell activations of our SmileCNN's last hidden layer. We demonstrate that the learned features have the excellent discriminative capability to train an SVM or AdaBoost classifier. Experiments on the GENKI4K database show that the proposed method can achieve promising performance in smile recognition. Pang et al. [41] provided a solution for visual target tracking tasks based on the CNN DL algorithm. On real-time visual tracking, the model obtained state-of-the-art performance. Another difficulty for video analysis is detecting human activity, which is currently being investigated in many studies. Ronao et al. [42] demonstrated an efficient and effective human activity detection system based on smartphone sensors that took advantage of the inherent properties of activities and ID time-series signals to identify them. On several experimental databases, this approach produced state-of-the-art outcomes that were previously unattainable.

## 3. Proposed Work

This research suggested a unique and novel architecture for evaluating facial expressions using a convolutional neural network implemented in a simulation environment. The process provided in our proposed model initially obtains a fresh raw image, referred to as image acquisition, from a variety of various datasets to ensure that our model is not biased toward any particular dataset. During this phase, our suggested model begins evaluating the selected image to detect the presence of a face. If it recognizes a face in the chosen image using a cascade classifier, it is passed to the 2nd phase for further preprocessing, where it is further refined. Image preprocessing is carried out during this phase, with several distinct stages being done, as illustrated in Figure 1. The facial expressions detected will be improved by utilizing various tools and techniques such as crop, rotate, flip, and stretch from the detected face. Afterward, the selected facial expressions are registered, and landmarks are recognized through normalization and magnification techniques. Micro and macro spotting are carried out on the landmarks chosen to extract the relevant and essential features in the following process phase. The final phase involves feeding the proposed CNN model with more data to forecast and categories the class.

## 4. Methodology

The proposed model comprises the following components used to perform various functionalities while evaluating the facial expression process from an image. These components are explained below.

### 4.1. Database

The Japanese female facial expression (JAEEE) dataset contains 213 samples of posture expression from 10 Japanese ladies, which are well-managed and laboratory-controlled. Six primary facial expressions are represented in three-quarters of each female image. These include smiles and scowls as well as angry, fearful, surprised, and disgusted looks. Since there are so few samples per participant and expression, the dataset poses a significant challenge. Laboratory-managed databases like the Extended Cohn-Kanade (CK+) are frequently consulted in the evaluation of FER systems. There are 593 video clips from 123 subjects in the dataset. Between 10 and 60 frames, the expressions change from neutral to ecstatic. There were 327 sequences from 118 people that were categorized with 7 basic emotion labels: contempt; anger; fear; happiness; surprise; sorrow; and disgust [43, 44].

### 4.2. Preprocessing

Unconstrained scenarios frequently feature differences in lighting, noise, head postures, and backgrounds that have little to do with facial expressions. Preprocessing is needed to align and standardize the visual semantic input before training the FER model on CNN. The following processes are included in the preprocessing phase, as outlined below.

1. Face detection is the foremost step in computer vision that locates a face area from the image. It states to find the face coordinates in the image, whereas localization refers to demarcating the extent of the face. The Viola–Jones (V&J) face detector is a classic and widely employed detection method [45].
2. In a deep learning-based FER system, data augmentation is essential. Whereas, large samples are needed to train the CNN model and provide generalizability to a specific recognition challenge. It is necessary to flip and crop the input images before they can be used in the machine learning process.
3. Face registration is a traditional preprocessing step in the face recognition task. Registration is done to align sample faces to a reference face. The subjects need not cooperate with data acquisition in the natural FER systems.
4. The eyes, mouth, nose, and eyebrows are all instances of facial landmarks that are used to locate and represent the most important parts of the face. We find the position of the subject's head and neck in the picture and note any distinctive features of their faces ROI.
5. The FER performance can be hampered by differences in illumination and head positions, which can result in considerable picture fluctuations. As a result, we present two common methods for normalizing faces to minimize these variations: normalization of lighting and head pose [46].

## 5. Convolutional Neural Networks

Deep learning methods use machine learning algorithms for forming high-level abstractions in emotions and pattern recognition in images and text [32]. The learning levels take the results of the previous levels as input, which are then converted and transformed into intuitions to train further and validate the classification model. The CNN model processes various types of information. The functionality of CNN creates complex layers to represent and process the complex data. Figure 1 shows the architecture of our face emotion detection FED model. The input of our model is a (48 × 48) grayscale image with some regularizations and optimization methods for the training system to understand and analyze the features. The output shows results in a single output class from seven emotions. The CNN network is composed of three convolutional layers, numbered C1 through C3, three MaxPooling layers, numbered P1 through P3, and four Relu activation functions, numbered R1 through R4. Additionally, as can be seen in Figure 1, all of these layers have complete connectivity between the input and output.

The C1 convolutional layer used filters on the input image, the size of the input image is 48 × 48, and learnable kernel/filters size used is 3 × 3 and produced 32 metrics with the size of (62 × 62). The results of the previous layer are used as input to the Relu activation layer, which fundamentally transforms the small range when the gradient is nonzero. The output Relu layer is used to the MaxPooling layer, which uses 2 × 2 learnable kernels. The output size of MaxPooling P1 matrices is (48 × 48). Similarly, these results are passed through the next convolutional layer C2 layer, with the same parameters. Finally, C3 and P3 layers use learnable kernels of size (3 × 3) and (2 × 2). Next, the flatten layer gives 4608 values; the first layer gives 2304 hidden units, and the other 1152. Lastly, the output layers generate seven classes, as shown in Table 1.

### 5.1. Hyperparameters

For the facial expression database, our suggested model utilizes a variety of hypermeters. Before going into the specifics of the model's performance on several databases, we briefly covered our training approach. Each dataset in our experiment was used to train our model; however, we made an effort to keep the architecture and hyperparameters consistent across models. From scratch, each model received 50 training epochs. We use a random Gaussian with zero and standard derivation to set the network weights in the beginning. Neuronal outputs were shaped by the activation function in the model, i.e., (Adam, AdaGrad, Nadam, and AdaMax). The output findings are shifted nonlinearly in response to their magnitude. By increasing in amplitude, signals spread and took on the shape of the final prediction of the network.

The entire demonstration of the CNN model is exceedingly complex and nonlinear because of the activation function. To reduce the model's error, the optimization functions Softmax, Softplus, Sigmoid, and Relu work together. In comparison to other optimization algorithms, Adam's performance appears to be the best with a learning rate of 0.003 and weight decay. With GPU, our model can be trained in 10 minutes on the FER database (using JAFFE and CK+). There are few samples; thus, the model can be completed within ten minutes. The regularization or shrining strategy was also employed to avoid overfitting the model, i.e., setting coefficients to 0. (dropout used between 0.1 and 0.4). Softmax activation is used for multiclassification in the dense layer after experimenting with a variety of combinations.

## 6. Results and Discussion

Experiments on two important facial expression recognition datasets are presented in this section, which includes the results of our model's evaluation. A brief overview of database concerns and challenges is presented, followed by an evaluation of the FER model's capabilities on two real-world datasets, CK+ and JAFFE, using a variety of hyperparameters. As FER work moves its focus to challenging environmental circumstances, many researchers are turning to deep learning apparatus in order to deal with challenges such as illumination variance, occlusions, nonfontal head positions identification bias, and recognition of low-intensity expressions. When using deep learning, it is essential to have a significant number of training examples available in order to accurately catch tiny expression-related bends. The primary challenge for deep FER systems is a deficiency in the quantity and quality of the training data.

We have split the dataset into 70% and 30% for the training and testing on both datasets.  Table 2 shows the comparison of the model on CK+ and JAEE datasets with epoch and batch size parameters, as table data depicted the performance of model outstanding with batch 128, 1024, and epoch 35, 50 on both databases. On the CK + dataset, our model achieved 97% testing accuracy with batch size 1024 and epoch 50 and a loss of 0.03. On the other hand, the JAFEE dataset with batch size 1024 and epoch 50 models recorded 65% and loss of 0.35.

Table 2 shows the experimental results on the CK + database's various basic and advanced parameters. The model is tested on 80 different combinations of parameters with distinct batch sizes and the number of epochs.

The approaches of regularization, optimization and activation are all used in this model. These are the activation functions that have been used: (Adam, AdaGrad, Nadam, Adamax, and hard Sigmoid), and the optimization procedures that have been used: (Softmax, Softplus, Sigmoid, and Relu). There is a difference between the regularization dropout ratio and (0.1 to 0.4). Softmax, Adam, and dropout values of 0.1 and 0.2 provide state-of-the-art accuracy for the FER model, which is the most accurate model currently available. When Softmax and Adam were used, the model claimed 94% testing accuracy with a dropout value of 0.1. This is depicted in Table 3.

Figures 2 and 3 illustrate the performance of a basic CNN model on CK+ in terms of loss and accuracy during testing on 50 iterations with 32 batch sizes. The accuracy of the simple CNN model is increasing concerning epochs. Similarly, the loss is displayed during the learning that is decreasing in each epoch.

Besides, Figures 4 and 5 show the training 97% and testing 70% accuracy on the CNN model using the JAFFE dataset and similarly, training loss of 0.07 and validation loss of 2.02.

Figure 6 shows that the model was able to learn from the CK + database [47].

## 7. Conclusions

The paper proposed a deep neural network (DNN) architecture for facial expression recognition (FER) based on convolutional neural networks (CNN). The CNN is one of the most representative network structures in the FER system and image processing in the deep learning field. The paper examined the emotional interpretation learning capacity of three distinct techniques, namely, activation, optimization, and regularization. Specifically, it has been noted that just two comparisons are completed with exceptional precision in terms of training, testing, and validation out of a total of 80 comparisons performed. There was a remarkable 0.1 difference in the model's accuracy when using Adam, Relu, and dropout data from other models. Using the FER2013 dataset, we ran a thorough experiment that yielded 97% training accuracy and 70% testing accuracy. A net loss of 0.05 and 2.01 is also shown. Using a simple CNN model, it is also discovered that the HOG operator's findings are ineffective when the image size is tiny and the image quality is unclear.

## Figures and Tables

**Figure 1:** Proposed system architecture.

**Figure 2:** CNN model CK+'s accuracy.

**Figure 3:** Loss of CNN model CK+.

**Figure 4:** Accuracy of the CNN model with CK + dataset.

**Figure 5:** Loss of the CNN model with JAFFE dataset.

**Figure 6:** Predication of model CK+.

**Table 1:** CNN configuration.

Layer (type)	Output shape	Param #
conv2d (Conv2D)	(None,128,128,6)	456
max_pooling2d (MaxPooling2D)	(None, 64,64,6)	0
conv2d_1 (Conv2D)	(None, 64,64,16)	2416
Activation (activation)	(None, 64,64,16)	0
max_pooling2d_1 (MaxPooling2)	(None, 32,32,16)	0
conv2d_2 (Conv2D)	(None, 30,30,64)	9280
max_pooling2d_2 (MaxPooling2)	(None, 15,15,64)	0
Flatten (flatten)	(None, 14400)	0
Dense (dense)	(None, 128)	1843328
Dropout (dropout)	(None, 128)	0
dense_1 (dense)	(None, 7)	903

**Table 2:** CNN results with CK+ and JAFEE.

Dataset	Epochs	Batch size	Test CNN Acc (%)	Test CNN loss
CK+	15	8	93	0.07
	20	16	94	0.06
	25	32	95	0.05
	30	64	94	0.06
	35	128	93	0.07
	40	256	96	0.07
	45	512	80	0.20
	50	1024	97	0.03
JAFFE	15	8	45	0.55
	20	16	48	0.52
	25	32	60	0.40
	30	64	49	0.51
	35	128	65	0.35
	40	256	42	0.58
	45	512	60	0.40
	50	1024	52	0.48

**Table 3:** Hyperparameters testing accuracy on the JAFEE dataset.

Activation	Optimization	Dropout	Testing accuracy
Softmax	Adam	0.1	0.94%
Softmax	AdaGrad	0.1	0.91%
Softmax	Nadam	0.1	0.92%
Softplus	Adamax	0.1	0.91%
Sigmoid	Adam	0.1	0.90%
Relu	Adam	0.1	0.93%
Relu	AdaGrad	0.1	0.91%
Relu	Nadam	0.1	0.90%
Relu	Adamax	0.1	0.90%
Softmax	Adam	0.2	0.95%
………	………	……….	……..
hard_sigmoid	Adamax	0.4	0.88%

## Data Availability

The data used in this research can be obtained from the corresponding authors upon request.
